# The Cellular State Determines the Effect of Melatonin on the Survival of Mixed Cerebellar Cell Culture

**DOI:** 10.1371/journal.pone.0106332

**Published:** 2014-09-03

**Authors:** Daiane Gil Franco, Regina P. Markus

**Affiliations:** Laboratory of Chronopharmacology, Institute of Bioscience, University of São Paulo, São Paulo, São Paulo, Brazil; University of Rouen, France

## Abstract

The constitutive activation of nuclear factor-κB (NF-κB), a key transcription factor involved in neuroinflammation, is essential for the survival of neurons *in situ* and of cerebellar granule cells in culture. Melatonin is known to inhibit the activation of NF-κB and has a cytoprotective function. In this study, we evaluated whether the cytoprotective effect of melatonin depends on the state of activation of a mixed cerebellar culture that is composed predominantly of granule cells; we tested the effect of melatonin on cultured rat cerebellar cells stimulated or not with lipopolysaccharide (LPS). The addition of melatonin (0.1 nM–1 µM) reduced the survival of naïve cells while inhibiting LPS-induced cell death. Melatonin (100 nM) transiently (15 min) inhibited the nuclear translocation of both NF-κB dimers (p50/p50, p50/RelA) and, after 60 min, increased the activation of p50/RelA. Melatonin-induced p50/RelA activity in naïve cells resulted in the transcription of inducible nitric oxide synthase (iNOS) and the production of NO. Otherwise, in cultures treated with LPS, melatonin blocked the LPS-induced activation of p50/RelA and the reduction in p50/p50 levels and inhibited iNOS expression and NO synthesis. Therefore, melatonin in vehicle-treated cells induces cell death, while it protects against LPS-induced cytotoxicity. In summary, we confirmed that melatonin is a neuroprotective drug when cerebellar cells are challenged; however, melatonin can also lead to cell death when the normal balance of the NF-κB pathway is disturbed. Our data provide a mechanistic basis for understanding the influence of cell context on the final output response of melatonin.

## Introduction

Nuclear factor kappa B (NF-κB) belongs to the Rel family that includes homo and heterodimers formed by p50, p52, RelA (p65), RelB and c-Rel. The dimers are sequestered in the cytoplasm by the inhibitory protein IκB. Various stimuli induce the complex IKK to phosphorylate the IκB that is degraded allowing NF-κB to translocate to the nucleus [1]. NF-κB is involved in the regulation of cell survival, proliferation, apoptosis and in inflammatory and immune responses [2]. In the brain, the most abundant NF-κB subunits are p50 and RelA [3]; however, c-Rel has also been detected [4]. The transcription factor NF-κB is constitutively activated in glutamatergic neurons and regulates physiological process such as cell migration, development, plasticity and synaptic transmission [5]–[7]. In addition, high levels of NF-κB are associated with neuropathological conditions and neurodegeneration [5], [8]. Therefore, because NF-κB represents a point of convergence of several pathways (including the activation of pro- and anti-apoptotic genes), it represents a potential pharmacological target for the treatment of neurodegenerative diseases.

Melatonin, an indolamine that is derived from serotonin and released at night by the pineal gland, contributes to cytoprotection that is mediated by G-protein-coupled membrane receptors or by the direct intracellular reduction of oxidative and nitrergic stress [9]–[11]. Melatonin has been shown to block the NF-κB pathway in murine macrophages [12], rat endothelial cells [13] and human neuroblastoma cells [14]. The inhibition of the nuclear translocation of NF-κB by melatonin blocks the expression of the inducible isoform of nitric oxide synthase (iNOS) and the synthesis of NO, conferring to melatonin a cytoprotective effect [12], [13]. Moreover, the administration of melatonin impairs the activation of NF-κB by cytotoxic substances and protects the liver and skeletal muscles by reducing the transcription of iNOS [15], [16]. For these reasons, the use of melatonin has been considered for the treatment or prevention of several neurodegenerative disorders [17], [18].

Not only the pineal gland can synthesize melatonin, but the brain tissue also express the key enzyme for the synthesis of melatonin, the arylalkylamine N-acetyltransferase (AA-NAT) [19]–[22] and there is evidence that this production is made by glial cells [22]–[24]. The importance of high levels of melatonin found in the central nervous system may be related to melatonin neuroprotective function [17]. The intracerebroventricular (icv) injection of lipopolysaccharide (LPS) in rats reduces nocturnal melatonin peak in the plasma and induces cell death in the hippocampus and in the cortex, but not in the cerebellum [22].

Cerebellar granule cell cultures represent a model of primary neuronal culture characterized by a basal level of NF-κB in the nucleus that is required for cell survival [3], [25]–[27]. This culture is maintained in a partially depolarized medium that elevates intracellular calcium levels [28], [29] and leads to proper NF-κB activation [30], [31]. Thus, a disruption in the normal balance of NF-κB activity (resulting in an increase or decrease in the nuclear content of this protein) may be related to cell damage [3], [6], [25]–[27]. Given the importance of this transcription factor for neuronal cell viability and the ability of melatonin to regulate NF-κB activity, we hypothesized that the modulation of NF-κB activity by melatonin in a naïve cerebellar granule cell culture or in a culture challenged with LPS (a stimulus known to activate the NF-κB pathway) could lead to cell damage or protection.

Our data confirm that, depending on the cellular context, melatonin leads to the activation or inhibition of the nuclear translocation of NF-κB, resulting in cell death or protection, respectively. As expected, melatonin impairs the LPS-induced activation of NF-κB, the expression of iNOS and the production of NO, all of which increase cell viability. In contrast, in naïve cultures, melatonin reduces cell viability by increasing the nuclear translocation of NF-κB, the expression of iNOS and the production of NO. Because NF-κB is an integrative point of convergence of several pathways involved in both physiological and pathogenic processes, elucidating the role of melatonin in different contexts will improve our understanding of its clinical output.

## Materials and Methods

### Animals

Wistar rats (male and female, 7–8 days old) from the animal facility of Institute of Biosciences - University of São Paulo (IB-USP) were used according to procedures approved by IB-USP Ethical Committee (CEUA/IB license number 110/2010) in compliance with the recommendation of the National Council on Experimental Animal Control (CONCEA).

### Drugs and reagents

Drugs and reagents purchased from Sigma-Aldrich (St. Louis, MI, EUA) included: trypsin; trypsin inhibitor; LPS from *E. coli* serotype 0127:B8; melatonin, 4-(2-hydroxyethyl)-1-piperazineethanesulfonic acid (HEPES); bis-acrilamida (N,N′-methylenebisacrylamide) and 3-(4,5-Dimethylthiazol-2-yl)-2,5-diphenyltetrazolium bromide (MTT). The following reagents were purchased from Santa Cruz Biotechnology (Santa Cruz, CA, USA): rabbit polyclonal antibody against iNOS (NOS2 (N-20):sc-651 TRITC) and NF-κB antibodies p50 (NLS)X sc-114X, p52 (K-27)X sc-298X, RelA (A)X sc-109X, RelB (C-19)X sc-226X, c-Rel (N)X sc-70X. The following reagents were purchased from GIBCO BRL Products (Grand Island, NY, USA): *Dulbecco's modified Eagles medium* (DMEM); fetal calf serum (FCS) and penicillin/streptomycin. Triton X-100 was purchased from Amresco (Solon, Ohio, USA). The following reagents were purchased from Invitrogen Life Technology (Carlsbad, CA, EUA): dithiothreitol (DTT), phenylmethanesulfonylfluoride (PMSF) and T4 polinucleotide kinase. Poly(deoxyinosinic-deoxycytidylic) acid sodium salt [poli(dIdC)] was purchased from Amersham Bioscience (Buckinghamshire, UK). Additional reagents were purchased from Bio-Rad (Richmond, CA, EUA) (acrylamide), Calbiochem (Darmstadt, Germany) (Nonidet-p40 (NP40), 1400W), Perkin Elmer (Boston, MA, USA) (Easy Tides: adenosine 5′- trifosfato, [γ^32^ P]), Promega (Madison, WI, USA) (Oligonucletotide consensus for NF-κB (5′-AGTTGAGGGGACTTTCCCAGGC-3′)), Molecular Probes (Eugene, OR, USA) (4-amino-5-methylamino-2′,7′difluorofluorescein diacetate (DAF-FM DA)) and IBL (Hamburg, Germany) (melatonin kit).

### Cerebellar cells culture

The rats were decapitated and their isolated cerebella were washed, cut into small pieces and incubated in 0.05% trypsin physiological solution (NaCl 120 mM, KCl 5 mM, KH_2_PO_4_ 1.2 mM, MgSO_4_.7H_2_O 1.2 mM, NaHCO_3_ 25 mM and glucose 13 mM; pH = 7.4) at 37°C for 40 minutes. The chemical dispersion was stopped with trypsin inhibitor (0.06%) and the cells that were isolated by mechanical dispersion were centrifuged (300 g, 5 min), plated in DMEM (13.4 g/L, FCS 10%, KCl 25 mM, NaHCO_3_ 44 mM, penicillin 50 U/ml/streptomycin 50 µg/mL; 5×10^5^–10^7^ cells/well) and maintained at 37°C, 5% CO_2_. Every 48 hours 50% of the medium was changed. Experiments were conducted on the seventh or eighth days of in vitro culture, and the medium was changed at least one hour before treatment.

The immunofluorescence staining using antibodies against MAP-2 (neuron marker), GFAP (astrocyte marker) and ED-1 (microglia marker) indicated that the cellular composition of the culture was 80–90% neurons, 10–15% astrocytes and 2–3% microglia. This culture is similar to that described by Kawamoto *et al.* [32] and Ohashi *et al*. [33].

### Experimental Protocols

The nuclear translocation of NF-κB was examined in cerebellar cells cultures challenged with LPS (100 ng/mL) for 15, 30 or 60 minutes in the presence or absence of melatonin (10 nM–1 µM). Cellular viability was assessed in cultures that were challenged with LPS (30–300 ng/mL) in the presence or absence of melatonin (10 nM–1 µM) for 24 hours. An iNOS activity inhibitor (1400W, 1 µM) was added to the culture 30 minutes before treatment with LPS or melatonin. The expression of iNOS was measured in cultures that were incubated with melatonin (10 nM–1 µM), LPS (100 ng/mL) or both for one hour. The production of nitric oxide was measured in cultures that were treated with LPS (100 ng/mL), melatonin (100 nM) or both for 24 hours. In all of the experiments, the control group was treated with a melatonin vehicle (ethanol 0.005%) and/or LPS vehicle (medium).

### Cell viability

Cell viability was assessed in cerebellar cell cultures using the MTT (a yellow tetrazole) method. MTT was added to cells at a final concentration of 0.005 g/mL and incubated for two hours to allow the reduction of MTT (which results in the formation of dark blue formazan crystals). The crystals were dissolved in dimethyl sulfoxide (DMSO) for 30 minutes in a shaker. Formazan production was measured by the change in absorbency at 540 nm using a microplate reader (SpectraMax 250, Molecular Devices, Sunnyvale, CA). Viability results were expressed as percentages of the absorbency measured in control cells.

### Electromobility-shift assay (EMSA)

Nuclear proteins were extracted from the cultures according to the method described by Ferreira *et al.* [34]. Briefly, the cultures were homogenized in lysis buffer (HEPES 10 mM, KCl 10 mM, EDTA 0.1 mM, DTT 1 mM, PMSF 0.1 mM), centrifuged (12000 g, 1 min) twice and resuspended in extraction buffer (HEPES 10 mM, KCl 500 mM, EDTA 1 mM, DTT 1 mM, PMSF 0.1 mM). After 15 minutes of incubation on ice and centrifugation (20,000 g, 5 min), the supernatant containing the nuclear proteins was collected in new microtubes and stored at −20°C. The total nuclear protein concentration was quantified at 280 nm using a ND-1000 spectrophotometer (Nanodrop, Wilmington, DE, USA). Six micrograms of protein were incubated in a final volume of 15 µL of binding buffer (Tris-HCl 10 mM pH 7.5; MgCl_2_ 1 mM; NaCl 50 mM; DTT 0.5 mM; EDTA 0.5 mM; glycerol 4%; poli-dIdC 1 µg) for 20 minutes at room temperature. Approximately 40,000 counts/min of double-stranded oligonucleotide probes containing the NF-κB consensus sequence (5′AGTTGAGGGGACTTTCCCAGGC) labeled with γATP-^32^P were added for 30 minutes at room temperature. The protein-DNA complexes were analyzed in non-denaturant 6% polyacrylamide gel at 150 V for 1.5 hours in tris-borato/EDTA buffer (TBE). After drying, the gel was exposed to a XAR-5 Kodak film (Rochester, NY, USA) for 48–72 hours at −80°C. Autoradiograms were analyzed densitometrically using the program ImageJ (Image Processing and Analysis in Java).

To identify NF-κB subunits, non-stimulated cells were incubated with 2 µg/mL of rabbit polyclonal affinity purified antibodies against p50, p52, RelA, RelB and c-Rel for 45 minutes at room temperature, before the addition of ^32^P-NFKB probe. EMSA was carried out as described previously.

### iNOS immunofluorescence

The expression of iNOS was measured according to an adapted protocol of Ferrari *et al.* [35]. The cells were washed with phosphate saline solution (PBS: NaCl 125 mM, Na_2_HPO_4_ 2 mM, NaH_2_PO_4_ 2 mM, KCl 5 mM) and fixed in methanol/acetone (1∶1, 15 min, 20°C). The cells were washed three times with phosphate saline and incubated for 30 minutes at room temperature with 0.2% Triton X-100 diluted in PBS. The preparation was incubated with anti-iNOS TRITC-conjugated antibodies [1∶50, Triton X-100 (0.2%)] and kept overnight at 4°C. The cells were then washed three times in PBS and the slides were mounted with PBS and glycerol (1∶1). The fluorescence was analyzed with an inverted confocal laser-scanning microscope equipped with a 40× oil-immersion objective (LSM 500, Carl Zeiss, New York, NY, USA) using the HeNe laser (543 nm) for excitation. To quantify the fluorescence, the LSM510 software (Carl Zeiss, LSM510) was used; only the granule cells (identified and differentiated from other cell types by their morphology) were considered. Five images containing 25–40 granule cells were randomly chosen and imaged as a 1024×1024-pixel frame; all of the other settings, including the pinhole, scanning speed and laser power, remained the same for all experiments. Inducible-NOS expression was evaluated as the percentage over the mean of the vehicle group.

### Nitric oxide

The level of NO was determined using the fluorescent indicator DAF-FM DA (5 µM), as previously described by Tamura *et al.* [36]. The cells were incubated in physiological solution (NaCl 140 nM, KCl 5 mM, MgCl_2_ 1 mM, CaCl_2_ 2 mM, glucose 5 mM, HEPES 5 mM, L-arginine 100 µM; pH 7.4) and treated for 24 hours with melatonin (100 nM) in the presence or absence of LPS (100 ng/mL). The control group received only the vehicle. The cells were incubated at room temperature for 50 minutes with 5 µM DAF-FM DA. The fluorescent compound was excited with an argon laser (488 nm) and the emitted fluorescence was measured at 515–530 nm using an inverted confocal laser-scanning microscope equipped with a 40× oil-immersion objective (LSM 500, Carl Zeiss, New York, NY, USA). The quantification of fluorescence was performed using the protocol described for iNOS expression. Nitric oxide levels were expressed as the percentage over the vehicle group.

### Statistical analyses

Data expressed as percentages of the vehicle were reported as the mean ± S.E.M. Results were compared by one-way analysis of variance (ANOVA) and the Newman-Keuls post-test.

## Results

The results of the MTT assay showed that LPS (30–300 ng/mL, 24 h) reduced the survival of cultured cerebellar cells by up to 40% (fig. 1A). Melatonin (0.1 nM–1 µM, 24 h) protected the cells against LPS (fig. 1B). Surprisingly, the control group incubated with melatonin (100 nM–1 µM, 24 h) experienced a 20% reduction in cell viability (fig. 1B), suggesting that, in the absence of LPS, melatonin itself can reduce cell viability. Because NF-κB is a common target for melatonin and LPS and cerebellar cells require a basal level of NF-κB activation for neuronal survival [3], we evaluated whether this central transcription factor involved in programming defense responses and neuronal survival could be involved in these conflicting effects of melatonin.

**Figure 1:** Dual effect of melatonin on the viability of cultured cerebellar cells. (A) Viability concentration-response curve for cells treated with LPS (30–300 ng/mL) incubated for 24 h; (B) Viability concentration-response curve for cells treated with melatonin (0.1 nM–1 µM) in the presence or absence of LPS (100 ng/mL), incubated for 24 hours. Each well contained 10^5^ cells at the beginning of the experiment. * p<0.05; **p<0.01 compared to control (n = 8–10 per point).

The transcription factor NF-κB is constitutively expressed in control cultures, as demonstrated by the results of the EMSA analysis (fig. 2A): antibodies against p50 and RelA identified p50/p50 and p50/RelA dimers, as the p50 antibody shifted both complexes but RelA shifted only the first complex. The other antibodies that were tested (p52, RelB and cRel) did not shift any complexes (data not shown).

**Figure 2:** Activation of nuclear factor-kappa B (NF-κB) in cultured cerebellar cells. (A) Super-shift assay performed with nuclear extracts from naïve cultured cerebellar cells incubated with antibodies against p50 and RelA subunits. The super-shift indicates the presence of the dimers p50/p50 and p50/RelA. (B) Time course for NF-κB activation by melatonin (100 nM) showing a transient reduction in the nuclear content of p50/p50 and p50/RelA followed by a significant increase in the nuclear content of p50/RelA (C) Concentration-response curve for melatonin (10 nM–1 µM, 15 min). (D) LPS (100 ng/mL, 15) induced NF-κB nuclear translocation in the presence or absence of melatonin (10 nM–1 µM, 15 min). For quantification the whole experiment present in graphs B, C and D was done in one gel, repeated 5 to 8 times. The values are expressed as percentage of the image detected in control conditions. * p<0.05% compared to control and # p<0.05 compared to LPS group (n = 5–8 per point). Symbols – squares: p50/RelA; triangles: p50/p50.

The incubation of the cultures with 100 nM melatonin induced a transient reduction in the nuclear level of p50/p50 and p50/RelA dimers during the first 15 minutes (fig. 2B). After 30 minutes of incubation, the nuclear levels of both NF-κB dimers were restored to their initial values; after 60 minutes of incubation, the nuclear content of p50/RelA (but not of p50/p50) was significantly increased. Because melatonin directly reduced levels of nuclear NF-κB within 15 min, we used this time interval to construct melatonin dose-response curves (fig. 2C). The maximal reduction in NF-κB content induced by melatonin (40%) was similar for both dimers; however, p50/RelA levels were reduced to a greater extent than p50/p50, indicating a specific sensitivity for each dimer. In summary, in cultured cerebellar cells melatonin produces a transient reduction in the nuclear content of both NF-κB dimers, followed by an increase of the p50/RelA nuclear activity above basal levels.

The addition of LPS (100 ng/mL, 15 min) significantly increased and decreased the nuclear content of p50/RelA and p50/p50, respectively (fig. 2D). Melatonin (10 nM–1 µM) blocked the LPS-induced nuclear translocation of p50/RelA but did not interfere with the reduction in levels of p50/p50, although the higher concentration of melatonin (1 µM) tended to increase levels of p50/p50 towards baseline levels. Therefore, in the presence of LPS, melatonin reduced NF-κB nuclear activity. The opposing effects of melatonin observed in naïve and LPS-treated cultures incubated for 60 minutes was in agreement with the dual effect on cell survival described in figure 1. The hypothesis of opposing effects was tested by evaluating phenotypic outputs (iNOS expression and NO production) and cell survival in the presence of the selective iNOS inhibitor 1400W.

The expression of iNOS in granule cells was evaluated by immunocytochemistry (fig. 3). The granule cells were identified by their rounded morphology and relatively small size (indicated by black arrows). Other cells with differentiated morphology (indicated by white arrow heads) were not quantified. Inducible-NOS was detected to be constitutively activated in the naïve group (fig. 3A). The addition of melatonin or LPS increased iNOS expression (fig. 3B, C, 4A). When melatonin was incubated with LPS, the expression of the enzyme was reduced to levels similar to those observed in the naïve group (fig. 3D, 4A).

**Figure 3:** Representative confocal microscopy image of immunocytochemistry for iNOS expression in cultured cerebellar cells. (A) Control, (B) incubation with 100 nM melatonin for 60 min, (C) incubation with 100 ng/mL LPS for 60 min and (D) incubation with melatonin + LPS. Black arrows indicate granule cells and white arrow heads indicate other types of cells (glial cells).

**Figure 4:** Quantification of the expression of iNOS. (A) LPS (100 ng/mL, 60 min) induced the expression of iNOS in the presence or absence of melatonin (30–300 nM, 60 min) (B) Time course of cells cultured with melatonin (100 nM), LPS (100 ng/mL) and melatonin + LPS. * p<0.05 and ** p<0.01 compared to control and # p<0.05 compared to LPS group (n = 4–6 per point). The number of cases refers to independent samples obtained in different days and from different cultures.

As predicted, LPS (100 ng/mL, 60 min) increased the expression of iNOS, while all of the concentrations of melatonin (30–300 nM) inhibited this effect of LPS (fig. 4A). The addition of melatonin in naïve cultures promoted a transient reduction in the expression of iNOS (30 min); however, after 120 minutes, iNOS levels were restored to levels slightly above basal levels (fig. 4B). Lipopolysaccharide induced an increase in iNOS expression above basal values within 30 minutes and this effect was blocked by melatonin (fig. 4B). Therefore, the effect of melatonin on iNOS expression was similar to that observed for the translocation of NF-κB.

As a result of the increase in iNOS expression, the incubation of cells with LPS (100 ng/mL, 24 h) or melatonin (100 nM, 24 h) led to an increase in the production of NO. In addition, melatonin blocked LPS-induced NO production (fig. 5A). The reduction in cell survival that was induced by LPS (100 ng/mL, 24 h) and melatonin (100 nM, 24 h) was not observed when the activity of iNOS was blocked by the selective antagonist 1400W (1 µM) (fig. 5B,C). Moreover, the blockage of iNOS activity increased cell survival in naïve cultures, indicating that the survival of this culture depends on the constitutive activity of iNOS.

**Figure 5:** The production of nitric oxide is responsible for melatonin- and LPS-induced cell death. (A) Quantification of NO production in cerebellar granule cells incubated with LPS (100 ng/mL, 24 h), melatonin (100 nM, 24 h) or melatonin + LPS. (B,C) Effect of the specific iNOS inhibitor (1400W, 1 µM) on the survival of granule cells cultured incubated with LPS (100 ng/mL, 24 h) or melatonin (100 nM, 24 h). * p<0.05%, ** p<0.01 and *** p<0.001 compared to control and # p<0.05 compared to LPS group (n = 3 per point).

## Discussion

Melatonin has been described as a cytoprotective and prosurvival agent that acts through both membrane receptor-dependent and independent mechanisms [11]. In this study, melatonin was confirmed to have a cytoprotective effect in cultures of cerebellum, which contains a majority of granule cells, incubated with LPS. Surprisingly, we also found that melatonin had a neurotoxic effect in cultures incubated without LPS.

The cerebellum, which is a target of melatonin G-protein coupled receptors [37]–[40], was used as a classical model to study the protective effect of melatonin against hyperbaric oxygen exposure [41], lipid peroxidation [42], [43], glutamate-induced neurotoxicity [44], aluminum exposition [45] and hypoxia [46]. Melatonin was shown to interfere with cerebellar tissue by inhibiting glutamate release [47], the transient outward flow of potassium [48], nicotinic currents [49] and the migration of granule cells [50]. Moreover, in rats the administration of LPS (icv) leads to the synthesis of melatonin in the cerebellum, but not in the hippocampus and cortex [22]. Even more, pinealectomy zeroed the content of melatonin in the cortex and hippocampus of LPS (icv) treated rats, while the level of melatonin in the cerebellum remains higher than those detected in animals killed at nighttime. The local synthesis of melatonin in the cerebellum was responsible for impairing cerebellar neuronal death.

The cerebellar granule cell culture requires elevated levels of potassium [28], [29], [51], [52] that increases intracellular calcium. The constitutive activity of NF-κB, that is necessary for maintaining cerebellar granule cell in vitro [3], [25]–[27], is consecutive of calcium entry into the cytosol [30]. An unbalance of NF-kB activity, in turn, leads to cell death [3], [7]. In this study, we examined the effect of melatonin on the viability of cerebellar cells in culture through modulation of the transcription factor NF-κB. Depending on the cellular context, the incubation of the culture with melatonin can result either in an increase or a decrease in the nuclear content of the p50/RelA subunit. This subunit contains the transactivating domain responsible for the transcription of the package of genes involved in cell defense, including the gene of iNOS. Therefore, an increase in the nuclear content of p50/RelA results in the production of NO and cell death.

We confirmed that cerebellar granule cells challenged by LPS express iNOS and produce NO [53]. Although we evaluated the expression of iNOS and NO production in granule cells, we can not ignore an indirect effect of LPS or melatonin through activation of glial cells in the culture. Despite the bidirectional interaction between glia and neurons is not yet well understood, it is known that the presence of glia in culture is needed to protect neurons [54]. The indirect effect of LPS was demonstrated in the pineal gland [55]. Although the main cell types of the pineal gland (pinealocytes, astrocytes and microglia) express TLR4, the production of TNF induced by LPS is mediated by microglia. The cytokine produced inhibits the synthesis of melatonin by pinealocytes.

The present study corroborated the results of several studies that demonstrated the beneficial effects brought about by the melatonin-mediated inhibition of NF-κB nuclear activity in vivo [15], [16], [56], [57] and in vitro [12], [13], [58]. The reduction in cellular viability observed in non-treated cells was most likely the result of an increase in the nuclear translocation of p50/RelA and therefore of the expression of iNOS and the production of NO resulting from a long-term incubation with melatonin. It is interesting to note that a melatonin-induced increase in reactive oxygen species (ROS) has been described in cancer cells [59]–[62] and appears to be associated with a reduction in tumor growth and proliferation. In addition, melatonin was shown to have a pro-oxidant effect that is mediated by an increase in NF-κB activity in a promonocytic cell line (U937) [63].

The present study shows that in non-treated cells melatonin inhibits the activation of NF-κB in the short-term, which tends to have a cytoprotective effect. The mechanism behind this effect likely involves the fine-tuned modulation of the NF-κB pathway by NO in a feedback loop. The NF-κB pathway is downregulated by an increased production of NO. The activation of neuronal NOS or pretreatment with NO donors inhibits the LPS- or tumor necrosis factor (TNF)-induced nuclear translocation of NF-κB [64]–[67]. The basic mechanism underlying this functional output involves the nitrosylation or nitration of key molecules in the NF-κB pathway. The S-nitrosylation of IKK impairs the activation of NF-κB [68]; in addition, the tyrosine nitration of RelA maintains this subunit in the cytoplasm [69] and the s-nitrosylation of p50 impairs the binding of homo and heterodimers to DNA [70], [71]. Nitric oxide also induces and stabilizes the NF-κB inhibitory protein IκBα [65]. Therefore, if the basal level of NO is reduced below a critical value, the loss of nitrosylation or nitration favors the activation of NF-κB and leads to an increase in iNOS expression and NO production. Our results therefore suggest that in naïve cultures melatonin reduces the nuclear level of NF-κB below basal values, resulting in a decrease in iNOS and NO that is sufficient to induce subsequent NF-κB activation. This increase only occurred with the transcriptional activator p50/RelA complex and not the inhibitory complex p50/p50, which results in the increased gene expression and reduced gene suppression. Thus, because iNOS expression is controlled by NF-κB, the addition of melatonin ultimately results in an increase in iNOS expression and NO production and a resultant reduction in cell survival. This hypothesis was confirmed by blocking melatonin-induced cell death with an inhibitor of iNOS activity. However, when cultured cerebellar cells are challenged by LPS, melatonin balanced the NF-κB activation generating cell protection.

In summary, we confirmed that melatonin can protect cerebellar cells that are challenged by a stimulus such as LPS; however, it can also induce a fatal loss in the normal balance of the NF-κB pathway. Thus, our data describe the mechanism behind the influence of the cell context on the final effect of melatonin.
